# Establishment of Narrow Root Fracture Models Using Modified Temperature Cycling Method and Diagnosis Using Different Cone-Beam CT Units

**DOI:** 10.1155/2022/3636795

**Published:** 2022-07-14

**Authors:** Jiahao Liang, Ziyang Hu, Dantong Cao, Ya Cao, Xin Xie, Antian Gao, Zhiyong Wang, Zitong Lin

**Affiliations:** ^1^Department of Dentomaxillofacial Radiology, Nanjing Stomatological Hospital, Medical School of Nanjing University, Nanjing, China; ^2^Department of Stomatology, Third People's Hospital of Danyang City, Danyang, China; ^3^Department of Oral and Maxillofacial Surgery, Nanjing Stomatological Hospital, Medical School of Nanjing University, Nanjing, China

## Abstract

**Aim:**

Using a modified thermal cycling method to establish narrow root fracture models and evaluate the diagnosis efficiency of them using four different cone-beam CT (CBCT) units. *Methodology*. Fifty-six intact teeth were selected, and the crowns of the teeth were embedded using general purpose acrylic resin. 50 root fracture models were established by soaking these teeth in liquid nitrogen and hot water cyclically; 6 teeth were used as the negative control. All the 56 teeth were scanned with the smallest voxel size of four different CBCT units (NewTom VGi, Planmeca Promax 3D Max, Kavo 3D eXam, and Soredex Scanora3D). 10 teeth were randomly selected, and the roots were sliced using slow-speed saw to obtain horizontal root sections. Scanning electron microscope (SEM) was used to measure the width of the fracture lines (FLs). The CBCT images were evaluated for the presence or absence of fracture lines. Accuracy, sensitivity, specificity, positive predictive value (PPV), and negative predictive value (NPV) were calculated for the diagnosis of FLs using the four CBCT units.

**Results:**

Fifty narrow root fracture models were successfully established, and 25 root sections with 45 FLs were acquired. The width of FLs was from 3.43 *μ*m to 143 *μ*m; 32.2% of the points had width under 25 *μ*m, while only 9.6% of them had width over 75 *μ*m. The accuracy was 0.41, 0.54, 0.41, and 0.30 for NewTom VGi, Planmeca Promax 3D Max, Kavo 3D eXam, and Soredex Scanora3D, respectively.

**Conclusions:**

The modified temperature cycling method is a simple and effective method to establish narrow root fracture models, and the diagnosis efficiency for these narrow fracture lines was quite poor using all the four different CBCT units.

## 1. Introduction

Root fracture is defined as a fracture of a tooth that involves the dentin, cementum, and pulp, and they may occur in any direction or orientation [1]. X-ray films enabled clinicians to visualize the roots which are surrounded by the alveolar bone and therefore provide important information for the diagnosis of root fractures and treatment planning. However, the conventional 2-dimensional X-ray films often could not give a definite diagnosis in clinical practice due to its disadvantages such as magnification, distortion, and anatomic superimposition. The recently widely used CBCT, due to its three-dimensional presentation of teeth with high spatial resolution, enhanced the accuracy of diagnosis of root fractures significantly and is being paid much attention to [2–6]. Although CBCT offers clear advantages over conventional X-ray films for the diagnosis of root fractures, the use of CBCT for the detection of root fractures remains controversial [7–9]. The complexity of fracture lines and the difference of CBCT units used in clinic are two important factors [10–12]. It is known that the ease of diagnosis will vary according to the extent of the fracture, and the detection of incomplete fractures and hairline-like fractures without obvious separation of the fractured fragments could be more difficult than obvious displaced root fractures. And different CBCT units have different voxel sizes, radiation doses, and reconstruction algorithms; these all may influence the quality of CBCT images and the diagnosis. To explore the influence of these two factors and establish a proper protocol of usage CBCT in clinic, many *in vitro* studies were performed. And the establishment of an artificial root fracture model with similar distribution with nature ones is the foundation of these researches. Mechanical methods were used to establish artificial vertical root fracture models in most previous studies [8, 12, 13], and the width of the fracture lines in those studies was uniform and much wider than the nature ones, especially wider than the ones at the initial stage.

The aim of this study was mainly 2-fold: firstly, we modified the thermal cycling method to establish narrow root fracture models which are more similar with the nature ones at the initial stage in clinic and secondly, compared the diagnosis efficiency of four different CBCT units with the smallest voxel size for these narrow root fracture lines.

## 2. Materials and Methods

### 2.1. Objectives

Fifty-six intact teeth were extracted with minimally invasive extraction due to orthodontic treatment plan or periodontal diseases at the Nanjing Stomatological Hospital, Medical School of Nanjing University. The inclusion criteria were no visual evidence of external cracks, craze lines, or fracture with the naked eye following extraction. The exclusion criteria were the presence of dental caries, root absorption, severe abrasion, wedge-shaped defects, and horizontal or vertical root fractures. This study was approved by the Ethics Committee of Nanjing Stomatological Hospital, Medical School of Nanjing University.

### 2.2. Establishment of Artificial Vertical Root Fracture Model

All 56 freshly extracted teeth were immediately immersed in saline solution (0.9% isotonic NaCl). Before establishing *in vitro* artificial root fracture models, the crowns of the teeth were embedded with general purpose acrylic resin (Unifast Trad, GC Corporation, Tokyo, Japan). Thereafter, 50 teeth were soaked in 100°C hot water for 1 min and then were quickly transferred into liquid nitrogen (-196°C) for 1 min; this procedure was repeated once there was one or more FLs observed on the surface of the root of the teeth with naked eyes. All the 50 teeth were finally confirmed to be positive root fracture models with the dental operating microscope (Carl Zeiss Meditec AG, S100/OPMI pico, Jena, Germany).

### 2.3. CBCT Image Acquisition and Evaluation

The 56 teeth were numbered and located on a piece of polystyrene foam and then scanned using the smallest voxel size of four different CBCT units (NewTom VGi, Planmeca Promax 3D Max, Kavo 3D eXam, and Soredex Scanora-3D). The details of the four CBCT units were showed in Table 1.

The CBCT images were viewed on a 29.7 in. screen MX300W LCD monitor (EizoNanao Corporation, Japan) and analyzed with inbuilt CBCT image analysis software of each unit (Planmeca Romexis Viewer for Planmeca Promax 3D Max, NNT Viewer for NewTom VGi and eXam Vision for Kavo 3D eXam, and OnDemand3D APP for Soredex Scanora3D).

Two observers (a radiological graduate student and an experienced radiologist) evaluated all images independently. If there was a hypodense line on axial images of teeth in at least 2 consecutive slices, the tooth was diagnosed as positive one. If a consensus could not be reached between the two examiners, a senior radiologist assisted in making the final decision. Before evaluation, calibration, including unified training on diagnostic standards of fracture line, was performed. After one week, the observers assessed all the images again to analyze the intraexaminer agreement.

### 2.4. Sample Preparation

#### 2.4.1. Acquirement of Root Sections with FLs

10 artificial root fracture teeth were randomly selected and stabilized in square mold filled with general purpose acrylic resin (Unifast Trad, GC Corporation, Tokyo, Japan) to embed the root of the teeth. Horizontal root sections with thickness of 2 mm were acquired from enamel-cemental junction to the apex of root using a slow-speed saw (Isomet, Buehler, Lake Bluff, IL, USA) under water cooling. Samples without visible fracture lines as well as complete fragmented were excluded. The process was shown in Figure 1. This procedure resulted in 25 root sections. All the 25 sections were numbered and marked, so facial, lingual, coronal, and apical sides could be identified. During all subsequent procedures, the sections were either stored in water or kept moist to prevent preparation shrinkage fracture or crack from dehydration.

#### 2.4.2. Measurement of Width of FLs Using SEM

The digitized images of the surface of each root section were captured with a magnification of 50x, 500x, or 1000x using a scanning electron microscope (SEM, S-3400N-II, Hitachi, Tokyo, Japan). Widths of FLs were measured at three points (S1, S2, and S3): S1 was near the root canal, S3 was in the outer cementum surface, and S2 was the middle point of S1 and S3 (Figure 2). These processes were operated by one operator in order to ensure the consistence of the measurements.

### 2.5. Statistical Analysis

Statistical analysis was conducted using the SPSS 22.0 software (IBM SPSS Statistics Base Integrated Edition 22, Armonk, NY, USA). The distribution of the FLs was analyzed. Accuracy, sensitivity, specificity, positive predictive value (PPV), and negative predictive value (NPV) were assessed in order to determine the diagnostic abilities of the four CBCT units. Kappa analysis was used to assess inter- and intraexaminer agreement.

## 3. Results

Twenty-five root sections with 45 FLs were acquired, and 135 points were selected and measured. The distribution of width of FLs was showed in Table 2. The widths of FLs were from 3.43 *μ*m to 143 *μ*m. 42.2% of the points had width under 25 *μ*m, while only 9.6% of them had width over 75 *μ*m. 10 of 45 FLs were S1 wider than S3, while the others were the opposite. Accuracy, sensitivity, specificity, PPV, and NPV of the four CBCT units were showed in Table 3. There was low inter- and intraexaminer agreement for the diagnosis, and the results were showed in Table 4.

## 4. Discussion

The diagnosis of root fracture can be extremely challenging in clinical practice. Because of the concealed location and atypical early symptoms, its exact diagnosis or prediction commonly requires abundant clinical experience and fine radiographic presentation. CBCT has been widely used in recent years for the detection of root fractures with relatively high accuracy and sensitivity benefit from its 3-dimensional image compared with 2-dimensional X-ray films [2, 5, 14]. However, the diagnosis of root fractures using CBCT was also controversial due to so many influenced factors existing (different widths and directions of fracture line, variables of CBCT units) [7, 15, 16]. To explore a more reliable and proper standard for using CBCT to diagnose root fractures, many *in vitro* studies were carried out [3, 10, 13]. And to establish an artificial root fracture model similar with the natural ones is the foundation of these studies.

There were two confusing concepts: crack and fracture. According to Rivera and Walton's review, the term ‘crack' implies an incomplete break in a substance. The term ‘fracture' implies a complete or incomplete break in a substance [17]. This means the crack lines could be narrower than fracture lines. And the fracture lines in the initial stage could be much narrower than those in the later stage. Therefore, the diagnosis of cracks or initial fractures could be more difficult than the diagnosis of later fractures.

There were mainly two categories of methods to produce crack or fracture lines in teeth: mechanical method and temperature control method. Mechanical methods were more commonly used to establish root fractures model. In Brady et al.'s study, incomplete and complete vertical root fractures were induced by inserting a sewing needle into the prepared canal and applying forces on the needle [8]. Makeeva et al. inserted posts into the root canal and gently tapped with a hammer to induce vertical root fractures [13]. Guo et al. produced vertical root fractures model by cutting the teeth using a diamond wire saw machine [12]. Lloyd et al. firstly used the thermal cycling method to produce cracks in teeth by using a thermal cycling apparatus allowing teeth cycled between hot and cold streams of water [18]. Wang et al. created cracks by exposure teeth into liquid nitrogen after hot water at 100°C [19]. In this study, artificial root fracture models were established by the modified thermal cycling method. The teeth were soaked in liquid nitrogen and hot water cyclically after their crowns were embedded with acrylic resin; this method avoids the teeth splitting completely and produced quite narrow fracture lines on the surface of the root.

The width of fracture lines produced by mechanical methods in previous study seems to be wider. In Makeeva et al.'s study, the width of the fracture lines ranged from 20 to 300, the mean width of fractures in the group 50–150 *μ*m was 96.3 ± 40.6 *μ*m, while for the group > 150 *μ*m the value was 230 ± 45 *μ*m, respectively [13]. In Guo et al.'s study, the width was 189-376 *μ*m for the wide group and 110-170 *μ*m for the narrow group and the mean width 279.5 ± 53.6 *μ*m and 140 ± 26.8 *μ*m, respectively [12]. However, in clinical practice, the width of fracture lines, especially for initial ones, is narrower than fracture lines induced by mechanical method. Huang et al. collected 37 extracted root fracture teeth and the width of fracture lines was between 10 and 1070 *μ*m (21.62% points was under 50 *μ*m) [20]. Our study established fracture lines with width between 3.43 *μ*m and 143 *μ*m, and 14.1% points was under 10 *μ*m, and 28.1% points was between 10 and 25 *μ*m. This was much narrower than the fracture lines induced by mechanical methods and could simulate the initial stage of fractures.

In the current study, although the smallest voxel size was used, the diagnosis efficiently for these narrow FLs was still quite poor using all the four different CBCT units. In our study, the highest accuracy was 0.54 which was obtained with Planmeca Promax 3D Max, and the highest specificity was also 0.54 which was obtained with Planmeca Promax 3D Max, which was much lower than the previous studies [5, 15, 21]. Considering that our models were nonendonotically treated, there were no artefacts resulting from endodontic filling. The width of most fracture lines was much lower than the voxel size of CBCT should be the main reason of the low diagnosis efficiency in this study. For narrow root fractures, the current CBCT units still have great limitation in the diagnosis (Figure 3). Therefore, it is possible that some root fractures may not be diagnosed at the time of initial presentation because the fractures are quite narrow.

Moreover, the fracture lines in our study were not consistent and uniform which was showed by SEM. This inconsistency at different points was similar with the condition in clinic [20], and fracture lines of 37 extracted vertical root fracture teeth showed inconsistent fracture space in Huang et al.'s study. This phenomenon indicated that the relationship between the width of FLs and voxel size of CBCT is more complicated than we assumed. If the FLs are much wider than the voxel size of CBCT, the detection of FLs could be of course easy, but if the width of FLs is close to or narrower than the voxel size, the condition could be sophisticated. The FL might be detected due to the wide part of it, and the FL may be presented as blurred and ambiguous on CBCT images.

## 5. Conclusions

In this study, we modified the thermal cycling method to establish artificial root fracture models; the widths of FLs were quite narrow and could stimulate the initial condition of fracture lines. The overall diagnosis efficiently for these narrow fracture lines was quite poor using current CBCT units. The relationship between the width of FLs and voxel size of CBCT is more complicated due to the complexity of fracture lines.

## Figures and Tables

**Figure 1:** (a) The crown of the teeth was embedded with general purpose acrylic resin. (b) Fracture line was observed on the surface of the root after soaking these teeth in liquid nitrogen and hot water cyclically. (c) The roots of the teeth were embedded with acrylic resin in a square mold. (d) The whole tooth was embedded with acrylic resin. (e) Horizontal root sections were acquired using a slow-speed saw. (f) The root sections with fracture lines were marked and numbered.

**Figure 2:** Widths of fracture lines measured at three points (S1, S2, and S3).

**Figure 3:** Example CBCT axial images of one tooth with root fracture scanned with the four CBCT units. (a, b) Fracture lines could be found on images scanned with 100 *μ*m voxel size of Planmeca Promax 3D Max and 100 *μ*m voxel size of NewTom VGi. (c, d) No fracture lines could be found on images scanned with 100 *μ*m voxel size of Soredex Scanora3D and 125 *μ*m voxel size of Kavo 3D eXam.

**Table 1:** Exposure parameters of four CBCT units.

CBCT units	FOV (cm)	Voxel size (*μ*m)	Tube voltage (kVp)	Tube current (mA)	Scan time (s)
NewTom	5∗5	100	110	7.48	6
Planmeca	5∗5	100	80	6.3	12.1
Soredex	5∗5	100	90	10	13.6
Kavo	8∗8	125	120	5.0	5

**Table 2:** Distribution of width of FLs using SEM.

	Width of fracture lines (*μ*m)					
	<10	10-25	25-50	50-75	75-125	125-150
No. of points	19	38	45	20	12	1
Frequency (%)	14.1	28.1	33.3	14.9	8.9	0.7

**Table 3:** Accuracy, sensitivity, specificity, PPV, and NPV of the four CBCT units.

	NewTom	Planmeca	Soredex	Kavo
Accuracy	0.41	0.54	0.41	0.30
Sensitivity	0.36	0.54	0.34	0.22
Specificity	0.83	0.50	1	1
PPV	0.95	0.90	1	1
NPV	0.14	0.12	0.15	0.13

PPV: positive predictive value, NPV: negative predictive value.

**Table 4:** The reliability of the 2 examiners with regard to FL detection.

	Intraobserver kappa	Interobserver kappa
NewTom	0.509	0.283
Planmeca	0.751	0.106
Soredex	0.509	0.211
Kavo	0.559	0.316

## Data Availability

The (.DICOM) data used to support the findings of this study were supplied by (Zitong Lin) under license and so cannot be made freely available. Requests for access to these data should be made to Zitong Lin (e-mail: linzitong_710@163.com).
